# PRDM14 is overexpressed in chronic pancreatitis prior to pancreatic cancer

**DOI:** 10.1002/2211-5463.12519

**Published:** 2018-09-17

**Authors:** Chiharu Moriya, Kohzoh Imai, Hiroaki Taniguchi

**Affiliations:** ^1^ Center for Antibody and Vaccine Therapy Research Hospital Institute of Medical Science The University of Tokyo Japan; ^2^ Research Hospital Institute of Medical Science The University of Tokyo Japan

**Keywords:** cancer stem cells, chronic inflammation, chronic pancreatitis, pancreatic cancer, PanIN, PRDM14

## Abstract

Pancreatic ductal adenocarcinoma (PDAC) is an aggressive and lethal cancer that is typically diagnosed at a later stage with metastases and is difficult to treat. Therefore, investigating the mechanism of PDAC initiation is important to aid early‐stage cancer detection. PRDM14 is a transcription factor that maintains pluripotency in embryonic stem cells and is overexpressed in several cancers. We previously reported that PRDM14 is overexpressed and regulates cancer stem‐like phenotypes in PDAC, and herein, we assess whether PRDM14 expression increases prior to tumorigenesis. Through immunohistochemistry analyses of clinical tissues, we detected PRDM14‐positive cells in precursor pancreatic intraepithelial neoplasia and chronic pancreatitis, which is a risk factor for PDAC, lesions. PRDM14 staining in chronic pancreatitis was as high as that in PDAC and cancer adjacent tissues. We induced pancreatitis in mouse models by cerulein injection, and observed that PRDM14 expression increased in chronic pancreatitis models but not in control or acute pancreatitis mice. Moreover, cerulein treatment increased PRDM14 expression in PK‐1 and AsPC‐1 pancreatic cancer cell lines. Our results suggest that inflammation increases the expression of PRDM14, which regulates cancer stem‐like phenotypes, and this occurs prior to PDAC initiation and progression.

**Abbreviations**
7‐AAD: 7‐amino actinomycin D
CHOP: C/EBP homologous protein
eIF2α: eukaryotic initiation factor 2 α‐subunit
ER: endoplasmic reticulum
FFPE: formalin‐fixed, paraffin‐embedded
GRP78: 78‐kDa glucose‐regulated protein
H&E: hematoxylin and eosin
IHC: immunohistochemistry
IPMN: intraductal pancreatic mucinous neoplasia
MCN: mucinous cystic neoplasia
NF‐κB: nuclear factor‐κB
PanIN: pancreatic intraepithelial neoplasia
PDAC: pancreatic ductal adenocarcinoma
ROS: reactive oxygen species
SP: side population
TMA: tissue microarray

Pancreatic ductal adenocarcinoma (PDAC) is one of the most aggressive and lethal diseases. This cancer presents aggressive phenotypes, such as progression, invasion, drug resistance, metastasis, and recurrence. Moreover, patients with PDAC do not present specific symptoms, and most of the time, the disease is diagnosed at a later stage with metastases 1. Therefore, screening tools to assist early‐stage PDAC detection and to histologically identify precursor cells and tissues are needed.

In PDAC, successive gene mutations and protein expression changes occur at various phases of tumorigenesis, including precursor conditions. Three premalignant precursor lesions of PDAC with different histological subtypes have been identified and are termed pancreatic intraepithelial neoplasia (PanIN), intraductal pancreatic mucinous neoplasia (IPMN), and mucinous cystic neoplasia (MCN) 1. PanIN is considered the most common precursor of PDAC, along with *KRAS* mutations, which occur in more than 90% of patients with PDAC and can be detected in the early PanIN stage 1, 2, 3.

Chronic pancreatitis is also considered a cause of pancreatic cancer 4 and a risk factor for PDAC, in addition to cigarette smoking, heavy alcohol intake, and diabetes mellitus 5. Chronic pancreatitis is commonly defined as continual inflammation of the pancreas that does not heal or improve, characterized by irreversible morphologic changes, such as the replacement of pancreatic acinar cells by fibrotic tissue. In contrast, acute pancreatitis, a sudden inflammation of pancreas that may result in life‐threatening complications, generally recovers completely and is not a risk factor for PDAC. The relation between cancer and chronic inflammation has been also suggested in other tissues. For example, hepatocellular carcinoma generally develops following chronic hepatitis with expression of hepatic progenitor cell markers, and the cancer stem cell phenotypes of hepatocellular carcinoma are inhibited by pharmacological inhibition of interleukin‐6 signaling, which is increased in chronic hepatitis 6, 7.

PRDM14 is a member of the PR domain‐containing family and a transcription regulator required for maintaining pluripotency in embryonic stem cells 8. PRDM14 is reported to be overexpressed in several cancers and related to cancer phenotypes 9, 10, 11. Recently, we reported that PRDM14 is overexpressed in PDAC tissues, compared to normal pancreatic tissues, and silencing the expression decreased cancer stem‐like phenotypes including side population (SP) cells, tumor formation, and liver metastasis 12. Interestingly, PRDM14 was also overexpressed in PDAC adjacent tissues, which were histologically non‐neoplasmic areas around the tumor, implying PRDM14 overexpression occurs at tumor origin and contributes to tumorigenesis 12. However, whether PRDM14 overexpression occurs prior to PDAC remains unknown.

In this study, we assessed the expression levels of PRDM14 in several pathological tissues, including PanIN and chronic pancreatitis. PRDM14 was overexpressed in chronic pancreatitis tissues as well as PDAC and cancer adjacent tissues. To estimate the relationship between PRDM14 overexpression and inflammation, we performed experiments using a cerulein‐induced chronic pancreatitis mouse model. Cerulein is an analogue of cholecystokinin, which shows high serum levels in patients with acute pancreatitis and is used for pancreatitis induction in a rodent model. Cerulein induces phenotypes of pancreatitis, such as amylase release, acinar cell death, and infiltration of inflammatory cells into the pancreas 13, 14, 15, 16. We also assessed PRDM14 expression in cerulein‐treated pancreatic cancer cell lines.

## Materials and methods

### Immunohistochemistry

Tissue microarray (TMA) slides containing pancreatitis and pancreas intraepithelial neoplasia were purchased from Biomax (Rockville, MD, USA; PA811, PA485, BIC14011). Mouse tissues were formalin‐fixed, paraffin‐embedded (FFPE), and sliced. IHC was performed as described previously 12. We used the following primary antibodies: human PRDM14 (ab187881) from Abcam Inc. (Cambridge, MA, USA) and mouse PRDM14 (#38965) from Signalway antibody (Pearland, TX, USA). The slides of mouse pancreatic tissues were also stained with hematoxylin and eosin (H&E) and Picro‐sirius red stain kit (ScyTek Laboratories, Inc., Logan, UT, USA) for collagen staining, according to manufacturer instructions.

By light microscopy, the tissue sections of TMA were scored semiquantitatively for PRDM14 staining, as described previously 12. Labeling scores were determined by multiplying the percentage of PRDM14‐positive cells per slide (0–100%) by the dominant staining intensity (0 = negative, 1 = trace, 2 = weak, 3 = intermediate, and 4 = strong). Resulting scores ranged from 0 to 400.

In this study, we used reported data on PRDM14 staining scores in normal pancreas, PDAC, and cancer adjacent tissues using TMA 12 to compare the expression levels with that in PanIN and chronic pancreatitis.

### Animals

Six‐week‐old female BALB/c mice were obtained from CLEA Japan, Inc. (Tokyo, Japan). Pancreatitis was induced referring to previous reports 4, 17. Chronic pancreatitis was induced by a single daily intraperitoneal injection of cerulein (0.1 mL of a 50 μg·mL^−1^ solution in saline, Bachem, Heidelberg, Germany) on five successive days. The pancreases were removed 3 days after the last cerulein injection. Acute pancreatitis was induced by 6‐hourly injections of cerulein in 1 day, and the pancreases were removed at 24 h after the first cerulein injection. The pancreases were used for IHC. All animal experiments were performed in accordance with the guidelines for the care and use of laboratory animals of the University of Tokyo and were approved by the Institutional Animal Care and Use Committee of the University of Tokyo.

### Cell culture

Two pancreatic cancer cell lines, PK‐1 and AsPC‐1 cells, were obtained and cultured as described previously 12. The cells were identified by the cell banks using short tandem repeat analysis. All cell lines were incubated at 37 °C in a humidified atmosphere containing 5% CO_2_.

### Cell treatment

Cells were incubated in culture medium in 6‐well plates for 24 h and were then stimulated with cerulein (100 nm) or brefeldin A (17.8 μm; #9972, Cell Signaling Technology Inc., Beverly, MA, USA) and collected after 24 h.

### Protein analysis by automated capillary electrophoresis, and immunodetection

Protein levels were quantified using an automated capillary electrophoresis and immunoassay system, Wes (ProteinSimple, CA, USA), as described previously 12. We used the following primary antibodies: PRDM14 (ab187881) and 78‐kDa glucose‐regulated protein (GRP78; ab21685) from Abcam Inc., C/EBP homologous protein (CHOP; #2895), GAPDH (#5174), eukaryotic initiation factor 2 α‐subunit (eIF2α; #5324), and phosphor‐eIF2α (Ser51, #3398) from Cell Signaling Technology Inc. The specificity of the PRDM14 antibody was confirmed previously by western blotting using knockdown cells 12.

### Analysis of SP cells

Isolation of SP cells was performed as described previously 12. Briefly, cells in suspension were incubated with Hoechst 33342 dye (Sigma‐Aldrich, St. Louis, MO, USA) with or without Reserpine (Sigma‐Aldrich), a multidrug transporter inhibitor. The cells were stained with 7‐amino actinomycin D (7‐AAD) (BD Pharmingen, San Diego, CA, USA) and analyzed using a FACSAria flow cytometer (BD Biosciences, San Jose, CA, USA).

## Results

### PRDM14 expression in precursor of PDAC and chronic pancreatitis

We assessed PRDM14 expression in PanIN (grade 1–3), which is considered the most common precursor of PDAC, by IHC using TMA (Fig. 1). PRDM14‐positive cells were detected in the PanIN structure. Although the PRDM14‐positive cells were detected in the lesions surrounding strong PRDM14‐positive PanIN, the periphery of PanIN lesions mostly showed no PRDM14 expression. Subsequently, we performed IHC using TMA of chronic pancreatitis, which is a risk factor of PDAC, and acute pancreatitis (Fig. 2A). PRDM14‐positive cells were detected in chronic pancreatitis tissues overall. In contrast, acute pancreatitis tissues did not show PRDM14 expression. The tissues were also scored for staining semiquantitatively and compared with the staining scores of normal pancreatic tissue, PDAC, and cancer adjacent tissues, which we previously reported 12 (Fig. 2B). PRDM14 expression score did not significantly increase in PanIN compared to normal pancreatic tissue, because PRDM14‐positive cells were few in the periphery. The staining score of chronic pancreatitis significantly increased to the level observed in PDAC and cancer adjacent tissues, while that of acute pancreatitis did not increase compared to normal tissue. The staining scores did not correlate with the PanIN grades (Table 1).

**Figure 1:** Expression of PRDM14 in PanIN. IHC was performed using a TMA slide that included PanIN. Representative IHC images for PRDM14 in PanIN tissues, grades 1–3. Tissues are shown with low and high staining intensity. Scale bars in image, 50 μm.

**Figure 2:** Expression of PRDM14 in pancreatitis. (A) Representative IHC images for PRDM14 in acute and chronic pancreatitis in TMA slide. Scale bars in image, 50 μm. (B) Staining scores and *P* values for PRDM14 in tissues, 13 normal pancreas, 115 PDAC, 36 cancer adjacent, 30 PanIN, six acute pancreatitis, and 58 chronic pancreatitis. Error bars in graphs represent mean ± SD. Student's *t*‐test: **P < 0.01, ns, not significant.

**Table 1:** Correlation of staining scores for PRDM14 in PanIN

PanIN grade	*n*	Core average	*P* value^a^
1	16	97.5	0.112
2	10	42.0	
3	3	56.7	

a One‐way ANOVA.

### PRDM14 expression in pancreatitis mouse model

Chronic inflammation is considered to be related to tumorigenesis 4, 7. Moreover, the staining score for PRDM14 was as high in chronic pancreatitis as in PDAC. Therefore, we investigated the relationship between PRDM14 expression and chronic pancreatitis. To assess the relation between inflammation and PRDM14 expression, we used a mouse model of pancreatitis, which was induced upon intraperitoneal injection of cerulein. We prepared both chronic and acute pancreatitis to assess whether continuous inflammation is needed for increased PRDM14 expression (Fig. 3). The pancreas of chronic pancreatitis had higher fibrosis, which was confirmed by staining with Sirius red, than that of control and acute pancreatitis (Fig. 4A), as reported previously 4, 17. On IHC analysis, PRDM14‐positive cells were observed in chronic pancreatitis models, but not in acute pancreatitis models and controls (Fig. 4A and B). These results suggested that chronic cerulein‐induced inflammation increases PRDM14 expression in pancreas of normal mice.

**Figure 3:** Pancreases with spleen of pancreatitis mouse models. Image of all pancreases with spleen of acute pancreatitis and chronic pancreatitis mice (*n* = 6 per group).

**Figure 4:** Pancreatitis mouse models. Acute and chronic pancreatitis was induced by intraperitoneal cerulein injection. Saline was used as control. (A) Representative images of the pancreases stained with H&E or Sirius red, and IHC for PRDM14 are shown. Scale bars in image, 200 μm. (B) High‐power magnification of IHC for PRDM14 of pancreas in chronic pancreatitis mouse models. The left panel is the enlarged image of the black box in the lower right panel in 3A. Scale bars in image, 50 μm.

### PRDM14 expression in cerulein‐stimulated pancreatic cancer cells

To assess the putative role of inflammation on PRDM14 expression in pancreatic cancer, pancreatic cancer cell lines, PK‐1 and AsPC‐1, were treated with cerulein. PRDM14 expression significantly increased upon cerulein treatment in both cell lines (*P* < 0.05) (Fig. 5). Additionally, endoplasmic reticulum (ER) stress is considered as one of the mechanisms of pancreatitis generation 18, and we previously reported that PRDM14 directly interacts with GRP78, which suggests a link between PRDM14 and ER stress 19. Thus, we also assessed the effect of an ER stress inducer brefeldin A. Although brefeldin A induced ER stress‐ and unfolded protein response (UPR)‐related downstream factors, GRP78, CHOP, and phosphorylated eIF2α, the drug did not increase PRDM14 expression (Fig. 5).

**Figure 5:** PRDM14 expression in pancreatic cancer cell lines. Pancreatic cancer cell lines, PK‐1 and AsPC‐1, were treated with cerulein and ER stress inducer brefeldin A. Expression levels of PRDM14, GAPDH, GRP78, eIF2α, phospho‐eIF2α, and CHOP in the cells were analyzed using Wes capillary electrophoresis system. GAPDH was used as a loading control. Expression levels of PRDM14 protein were normalized to that of GAPDH and plotted as fold changes relative to control. Error bars represent the mean ± SD of triplicate samples. Student's *t*‐test: **P < 0.01, *P < 0.05, ns, not significant.

We have previously reported that PRDM14 regulates cancer stem‐like phenotypes in pancreatic cancer cells 12. Therefore, we assessed the number of SP cells, a cancer stem‐like phenotype, in cerulein‐treated cancer cell lines. SP cells very slightly increased in AsPC‐1 cells (*P* < 0.01), but did not significantly change in PK‐1 cells (Fig. 6).

**Figure 6:** Side population cells in cerulein‐treated PK‐1 and AsPC‐1 cells. SP cells in cerulein‐treated PK‐1 and AsPC‐1 cells analyzed by flow cytometry using Hoechst 33342 dye. Reserpine, a multidrug transporter inhibitor, was used as a control for SP. Error bars in graphs represent mean ± SD of triplicate samples. Student's *t*‐test: **P < 0.01, ns, not significant.

## Discussion

Pancreatic ductal adenocarcinoma is an aggressive and lethal disease, and screening tools for early‐stage detection are needed. We previously found that PRDM14 was overexpressed in PDAC and cancer adjacent tissues, compared to normal pancreatic tissues, and regulates cancer phenotypes 12. Therefore, in this report we assessed PRDM14 expression in precursor lesions of PDAC and chronic pancreatitis, which is a risk factor of the disease. PRDM14‐positive cells were observed in both PanIN and chronic pancreatitis (Figs 1 and 2A). Interestingly, the staining score for PRDM14 in chronic pancreatitis was as elevated as that observed in PDAC and cancer adjacent tissues (Fig. 2B).

Recent studies have demonstrated that inflammation relates to various processes of tumor formation, including cancer initiation in early lesions, progression, and metastasis. Chronic inflammation, a repeat of injury and healing processes, is considered a trigger of tumorigenesis in several tissues 7, 20. In the pancreas, chronic pancreatitis is a risk factor of PDAC and is reported to initiate precursor lesions and assist the progression of such lesions to PDAC. Cerulein‐induced chronic pancreatitis causes PanIN and invasive pancreatic cancer formation in KRAS‐mutant mice, in which they are not formed by mutation alone 4, 21. Inflammatory responses induced by tumor‐associated immune cells cause cancer cells to metastasize and migrate through the epithelial–mesenchymal transition 21, 22. Various inflammatory modulators, such as prostaglandin E2, have been shown to facilitate tumor progression, while anti‐inflammatory agents have been found to inhibit tumor growth 23, 24. Furthermore, the relationship between inflammation and cancer stemness is also being gradually elucidated through the association between inflammation and cancer initiation, metastasis, and EMT. Prostaglandin E2 is also reported to enhance cancer stem‐like phenotypes and increase proliferation of CSCs 25, 26, 27. A cancer stem cell marker DclK1, which is also reported to be expressed in PanIN and facilitate tumor progression in KRAS‐mutated mice and human pancreatic cancer, was upregulated by cerulein 28. PRDM14 is known to relate to pluripotency in ES cells and to cancer stem‐like properties in breast and pancreatic cancers 8, 11, 12. In this study, PRDM14‐positive cells were detected in PanIN and chronic pancreatitis (Figs 1 and 2A) in addition to PDAC tissues 12. Moreover, chronic pancreatitis induced by cerulein increased PRDM14 expression in the pancreases of normal mice (Fig. 4). We have so far been unable to confirm whether PRDM14 expression is controlled at the transcriptional level and cannot exclude the possibility that the protein turnover is regulated. However, these findings support the participation of chronic inflammation in inducing cancer stemness prior to tumor progression. On the other hand, acute pancreatitis did not increase PRDM14 expression in normal pancreatic tissue (Fig. 4) indicating the important effect of chronic inflammation on cancer initiation and tumorigenesis.

Several mechanisms of pancreatitis generation have been identified, such as activation of nuclear factor‐κB (NF‐κB) 29, ER stress 18, 30, and autophagy signaling in acinar cells 31. Cerulein, which we used in this study, is considered to produce reactive oxygen species (ROS), which induce NF‐κB and to activate inflammasomes, leading to inflammation 13, 32. Repeat injection of cerulein is also reported to induce chronic ER stress as well as chronic pancreatitis 18, 32. Previously, we reported the direct binding and cooperation of PRDM14 with GRP78, which is a heat‐shock protein upregulated after ER stress, suggesting a relationship between ER stress and PRDM14 19. A single treatment with ER stress inducers, which increased GRP78, did not increase PRDM14 expression in pancreatic cancer cell lines (Fig. 5). On the other hand, cerulein treatment increased PRDM14 expression without increasing GRP78 expression. Although transfection of the binding partners did not also affect each protein's expression 19, these results indicate that upregulation of PRDM14 expression by inflammation in pancreatic cancer cells required other pathways than ER stress.

We previously reported that inhibition of PRDM14 expression decreases cancer stem‐like phenotypes, including SP cells, in pancreatic cancer cells 12. Although cerulein increased PRDM14 expression in pancreatic cancer cell lines, it did not increase the number of SP cells (Figs 5 and 6). Because PRDM14 expression is already elevated, additional increase may have minimal effects. Furthermore, repeated cerulein treatment on successive days was needed to increase PRDM14 expression in the pancreas of normal mice, and 1‐day treatment was not sufficient for increase (Fig. 4). However, single stimulation with cerulein was enough to increase PRDM14 expression in pancreatic cancer cell lines (Fig. 5). A normal pancreas may require repeated inflammation for induction of PRDM14 overexpression, while a single inflammation may be enough for already transformed pancreatic cancer cells. Although inflammation increased PRDM14 expression in PDAC cells without enhancing cancer stem‐like phenotypes, inflammation may contribute to maintain the overexpression and tumor phenotypes in the cancer. Anti‐inflammatory reagents have been reported to inhibit tumor growth and cancer stem‐like phenotypes 23, 25, 28, 33. PRDM14 expression may also be associated with anti‐inflammatory effects on tumor phenotypes.

Our results revealed that cerulein‐induced chronic pancreatitis increased PRDM14 expression in normal mice. Cerulein alone is not enough for tumorigenesis, and the combination with other factors is needed. For example, cerulein induces pancreatitis, but not PDAC, in mice without KRAS mutation, and induces pancreatitis, PanIN, and PDAC in mice with genetic KRAS mutations. To investigate the effects of PRDM14 expression induction by chronic pancreatitis on tumorigenesis, more experiments using transgenic mice, such as those harboring KRAS mutations and PRDM14 knockouts, should be performed in the future. If PRDM14 knockout reduces either inflammatory responses or the formation of PanIN and PDAC, targeting PRDM14 expression may be useful treatment strategy against the early lesions prior to PDAC.

PRDM14 is overexpressed in PDAC and regulates cancer stem‐like phenotypes. In this study, we detected PRDM14‐positive cells in PanIN and chronic pancreatitis. Using pancreatitis mouse models, we observed that cerulein‐induced chronic inflammation on successive days increases PRDM14 expression in the pancreas of normal mice. Moreover, cerulein also increases PRDM14 expression in pancreatic cancer cells. Taken together, PRDM14 overexpression may be triggered by chronic pancreatitis prior to PDAC and regulate tumor initiation and progression.

## Author contributions

CM and HT designed the experiments. CM performed the experiments, analyzed and interpreted data, and wrote the manuscript. KI supervised the research. All authors read and approved the manuscript.
